# A New Arbiter PUF for Enhancing Unpredictability on FPGA

**DOI:** 10.1155/2015/864812

**Published:** 2015-09-30

**Authors:** Takanori Machida, Dai Yamamoto, Mitsugu Iwamoto, Kazuo Sakiyama

**Affiliations:** ^1^The University of Electro-Communications, 1-5-1 Chofugaoka, Chofu-shi, Tokyo 182-8585, Japan; ^2^Fujitsu Laboratories Ltd., 4-1-1 Kamikodanaka, Nakahara-ku, Kawasaki-shi, Kanagawa 211-8588, Japan

## Abstract

In general, conventional Arbiter-based Physically Unclonable Functions (PUFs) generate responses with low unpredictability. The *N*-XOR Arbiter PUF, proposed in 2007, is a well-known technique for improving this unpredictability. In this paper, we propose a novel design for Arbiter PUF, called *Double Arbiter PUF*, to enhance the unpredictability on field programmable gate arrays (FPGAs), and we compare our design to conventional *N*-XOR Arbiter PUFs. One metric for judging the unpredictability of responses is to measure their tolerance to machine-learning attacks. Although our previous work showed the superiority of Double Arbiter PUFs regarding unpredictability, its details were not clarified. We evaluate the dependency on the number of training samples for machine learning, and we discuss the reason why Double Arbiter PUFs are more tolerant than the *N*-XOR Arbiter PUFs by evaluating *intrachip variation*. Further, the conventional Arbiter PUFs and proposed Double Arbiter PUFs are evaluated according to other metrics, namely, their uniqueness, randomness, and steadiness. We demonstrate that *3-1 Double Arbiter PUF* archives the best performance overall.

## 1. Introduction

### 1.1. Background

Nowadays, many products related to our daily life are being connected to the Internet and controlled by computers. Thus, machine-to-machine communication is an increasingly common phenomenon. Secure authentications between these machines are needed for security,* for example*, to avoid fake integrated circuits. Physically Unclonable Functions (PUFs) [1, 2] have been proposed as a solution to this problem [3]. Authentication utilizing PUFs can provide the protection of an authentication chip on a device, and intellectual property core protection for field programmable gate arrays (FPGAs) [4, 5].

PUFs are physical functions that output a unique value as a response to an input known as a challenge. The response reflects the manufacturing variation of the physical unit. A verifier stores challenge-response pairs (CRPs) to test the authenticity of the so-called prover. The stored responses in the verifier are compared with the responses provided by the prover according to the same challenge. This comparison of responses enables the verifier to confirm whether the prover is genuine. This authentication mechanism is considered secure insofar as it is difficult to copy the manufacturing variation of the PUF. Because PUFs can be implemented with comparatively small circuits, they facilitate lightweight authentication.

PUFs can be implemented not only on an application specific integrated circuit (ASIC) [6], but also on an FPGA [7]. FPGAs are embedded in various products that require both customizability and security, because synthesizing FPGAs is programmable. For low-volume manufacturing, it is relatively less expensive to produce a product with an FPGA than a product with an ASIC.

Many types of PUFs have been proposed. The authors of [8] categorize them into two types: memory-based and delay-based PUFs. We focus on Arbiter-based PUFs, a variety of delay-based PUFs. Delay-based PUFs use delay-time information from the signal propagation in the circuit. The basic concept of an Arbiter PUF was described in 2002 [9]. They are based on the delay-time difference between two signals. Arbiter PUFs that consist of symmetrically located wires and selectors were proposed in 2004 [10, 11], and they were evaluated using various metrics. Other authors categorize PUFs into strong PUFs and weak PUFs [5]. On the one hand, the former PUFs have a relatively large challenge space;* that is*, they can use many challenges, making them suitable for the device identification and authentication. The relation between challenges and responses is too complex to be accurately predicted. Previous work also suggests that the responses from some of these PUFs can be predicted by modeling attacks based on machine learning, which uses a mathematical model established by authorized CRPs. Consequently, the Arbiter PUF was once considered a candidate for a strong PUF but has since been found to be vulnerable to such modeling attacks [12, 13]. On the other hand, weak PUFs have either no challenge space or one that is relatively small. Weak PUFs can be used for key generation or for some cryptographic protocols on a device because it often generates stable responses in repeated measurements [14, 15].

In this paper, we discuss secure Arbiter PUF implemented on FPGA. (Parts of this paper are based on [16–18]. This paper newly discusses optimal implementations for high tolerance against machine-learning attack, along with high uniqueness and steadiness.)

### 1.2. Motivation and Contribution

The authors of [19] proposed the *N*-XOR Arbiter PUF that uses the XOR *N* responses from the *N* Arbiter PUFs implemented on the same chip to decrease the predictability of the responses. In this paper, we introduce a novel Arbiter PUF,* Double Arbiter PUF*, which was originally proposed as a technique for generating highly unique responses [16]. We expect that our Double Arbiter PUF will be a valid approach for enhancing unpredictability even on FPGAs that have wiring problem (see Section 3, below). The authors of [17] proposed* 2-1 Double Arbiter PUF* whose response is obtained by two XORing responses from the Double Arbiter PUF.* 3-1 Double Arbiter PUF* was also proposed in [17]. This PUF has a third building block, and its response is generated by six XORing responses from these building blocks. Although the authors of [18] considered the tolerance of conventional Arbiter PUF and Double Arbiter PUFs to machine-learning attacks, they did not compare them with the *N*-XOR Arbiter PUF. Further, there were no results that showed a dependency on the number of training samples in [18]. We newly evaluate *N*-XOR Arbiter PUFs and Double Arbiter PUFs according to this tolerance, by using between 100 and 1,000 training samples. In order to clarify the reason why the Double Arbiter PUF is more effective than the conventional *N*-XOR Arbiter PUF at XORing responses for adding the unpredictability, we evaluate these PUFs according to* intrachip variation*, a metric defined in this paper. Our experimental results show that the intrachip variation of Double Arbiter PUFs is much higher than that of the conventional Arbiter PUF and that its tolerance against machine-learning attacks is also relatively high, regardless of number of training samples. In particular, it is difficult to predict responses from the 3-1 Double Arbiter PUF because the prediction rate of the responses for randomly chosen challenges is approximately 57%, and this is close to 50%, random guess.

XORing responses from multiple PUFs within the same chip can be also expected to increase the interchip difference among chips that has been evaluated according to* uniqueness* [20]. We introduce the results from [17] regarding uniqueness and confirm that the uniqueness of the Double Arbiter PUFs is almost ideal and much higher than that of conventional *N*-XOR Arbiter PUFs. In this paper, we newly propose* 4-1 Double Arbiter PUF* that has a fourth building block. The response from this PUF is generated by more XORing responses than the 3-1 Double Arbiter PUF. From our experimental results, we demonstrate the proposed PUF's tolerance to machine-learning attacks and its uniqueness, both of which are comparable to the 3-1 Double Arbiter PUF. A high level of stability in the responses is also needed when repeating the same challenge for the device authentication using PUFs, a metric referred to as* steadiness* [20]. Because our results show low steadiness in the 4-1 Double Arbiter PUF, we conclude that the 3-1 Double Arbiter PUF is the most suitable PUF for device authentication.

Our contributions are summarized as follows:

(i) We show that the 3-1 Double Arbiter PUF has much higher tolerance to machine-learning attacks than the conventional *N*-XOR Arbiter PUF.
(ii) We also conclude that the 3-1 Double Arbiter PUF demonstrates the best performance from among the introduced PUFs, in terms of tolerance, uniqueness, and steadiness.

### 1.3. Organization of This Paper

Section 2 shows the related work: the structure of conventional Arbiter PUFs, the reason why conventional Arbiter PUFs are vulnerable to machine-learning attacks, and their countermeasures. In Section 3, we introduce the Double Arbiter PUFs as an alternative countermeasure. Our experimental environment and the metrics for our evaluation, including the intrachip variation, are described in Section 4.  Section 5 compares the conventional Arbiter PUF with the Double Arbiter PUF, in terms of their tolerance to machine-learning attacks.  Section 6 provides the results from a performance evaluation based on [17] and discusses the feasibility of the introduced PUFs for device authentication. Finally, we conclude the paper in Section 7.

## 2. Related Work

### 2.1. Arbiter PUF

The Arbiter PUF, proposed in [10, 11], consists of selector pairs connected in a series and an Arbiter (an SR-Latch is used, as shown in Figure 1) that determines its response, as shown in Figure 1. First, an input signal is supplied to the first left and right selectors at the same time. The genetic idea behind Arbiter PUFs is to race the delay times between the two signals. The two signals propagate through various routes depending on the value of the challenges. These routes are determined by an *n*-bit challenge that is given as the selection input for the selector pairs. The (*i* + 1)th challenge bit *c*_*i*_ out from the *n*-bit challenge corresponds to the selection inputs for the (*i* + 1)th selector pair, where *i* = 0,1,…, *n* − 1. When *c*_*i*_ = 1, two output signals from the *i*th selector pair are crossed and supplied to the selection inputs for the (*i* + 1)th selector pair. When *c*_*i*_ = 0, the two signals are directly supplied to the selection inputs for the (*i* + 1)th selector pair. A 1-bit response 1/0 is determined by which signal reaches an Arbiter faster than the other. The size of the challenge space is 2^*n*^, such that 2^*n*^ patterns of the propagation delay time can be organized. Physically, the wire length of the two lines should be the same.

### 2.2. Machine-Learning Attacks for Arbiter PUFs

In this section, a framework for machine-learning attacks with a delay model is explained by referring to [12, 13], and we discuss how responses from the Arbiter PUF can be predicted with machine learning.

The basic concept for machine learning is as follows. Each route through which two signals traverse is determined by a challenge for the Arbiter PUF, and a response is determined by the delay-time difference of the signals. Let **w** be a model of the delay times for an Arbiter PUF. Let **φ** be a model extracted from a challenge for this Arbiter PUF, and let *r* be a response. Because a response is determined with a sign of the delay-time difference between two signals, the response can be expressed as

(1) $$\begin{array}{c} r=\mathrm{sgn}\left(\;w^{T}\varphi \;\right), \end{array}$$

where sgn is a sign function and **w** ^*T*^ denotes the transposed **w**. Because it is difficult to know the delay times **w**, the pair for a response *r* and a model for the challenge **φ** is given, and a model for the delay times is constructed.

The procedure for machine learning consists of two phases, a training phase and a classification phase, as shown in Figure 2. During the training phase, several pairs of challenges *c* and responses *r* from the target Arbiter PUF are initially prepared. Then,* feature extraction* is performed. Challenge *c* is transformed in order to simplify the machine learning process. The procedure of this challenge transformation from *c* to **φ** is as follows. Let *c*_*k*_ be the *k*th bit of a challenge, where *k*  ( = 1,2,…, *n*) denotes the length of the challenge. Let *φ*_*i*_ be the *i*th bit of the transformed challenge, where *c* ∈ {1,0}^*n*^, *i* = 1,2,…, *n* + 1, and **φ** ∈ {1, −1}^*n*−1^. The challenge model is **φ** expressed as

(2) $$\begin{array}{c} \varphi_{i}=\left\{\begin{array}{cc} \overset{n}{\underset{k=i}{\prod }}\left(1-2c_{k}\right) & \left(i=1,2,\ldots ,n\right)\\ 1 & \left(i=n+1\right). \end{array}\right. \end{array}$$

After feature extraction, a model for the delay times **w** is constructed, depending on the pair of the challenge model **φ** and the response *r*.

A different challenge *c*′, whose response is unknown, is provided during the classification phase. After feature extraction from *c*′ to **φ**′, the response *r*′ is predicted by using the model for the delay times **w** constructed during the training phase, as follows:

(3) $$\begin{array}{c} r^{\prime }=\mathrm{sgn}\left(\;w^{T}\varphi^{\prime }\;\right). \end{array}$$

The response *r*′ is the output from machine learning, and we can evaluate whether *r*′ is equivalent to the response obtained from the Arbiter PUF, given *c*′.

Feature extraction must be more fully elaborated. First, we explain the relationship between *c* and **φ** by using the example shown in Figure 3. Figure 3 shows one part of an Arbiter PUF, including the selector pairs and wires to which a challenge from the (*n* − 3)th to the *n*th is given. The dashed red and solid black lines refer to an example of two paths when the challenge *c*_*k*_ from the (*n* − 3)th to the *n*th is “0110.” Then, we focus on the wire illustrated as a dashed line out of the two wires. The value of the challenge model **φ** shows which signal is located in the right position between selector pairs. Suppose that a signal through the wire (the dashed line) has a long delay time at the output of the (*n* − 4)th selector pair. If we use the challenge model **φ**, we can easily recognize which signal (whether the dashed or solid line) is located in the right position at the output of the last selector pair.

Suppose that there is a pair of challenges, where one is chosen randomly and the other involves a 1-bit flip of this challenge. Although the Hamming distance between the pair of challenges is small,* that is*, insofar as the challenges are similar, the pair of responses related to the pair of challenges can have different values, because the position of the signal through the dashed or solid line at the output of the last selector pair is exchanged. By contrast, when the same pair of challenge model vectors **φ** is given, namely, the randomly chosen vector and the 1-bit flipped vector, the pair of responses can have the same value, because the position of the signal is not exchanged. It is worth noting that the signal through the dashed and solid line with the original challenge has a total delay time similar to that of the signal with the similar challenge. This consideration is important to Section 5.1 when discussing a challenge model for a Double Arbiter PUFs.

### 2.3. *N*-XOR Arbiter PUFs for Unpredictability

Previous work [19] has proposed the *N*-XOR Arbiter PUFs as a countermeasure against machine-learning attacks. The authors of [19] aimed to obfuscate the response by XORing *N* responses obtained from *N* Arbiter PUFs on the same chip. Figures 4 and 5 show the structures for the 2- and 3-XOR Arbiter PUF, respectively.

## 3. New Arbiter PUFs for Unpredictability

In this section, we introduce the Double Arbiter PUF [16] as another approach to enhance the unpredictability of responses. The Double Arbiter PUF was originally proposed in [16] as a technique for increasing variety of responses among chips.

In general, it is difficult to implement two wires of exactly the same length (so-called equal-length wiring), not only on FPGAs but also on ASICs. With two wires of unequal length, the two signals through these wires will have obvious differences in delay times. Suppose that we compare two signals through specific paths, where the length of the wires is unequal in an Arbiter PUF. If this delay time is longer than the delay time based solely on the physical variation of the devices, the response from the chips will be the same. That is, there will be no difference in the responses of the devices. Further, because it is easy to predict these responses, this wiring problem is pertinent to the unpredictability of the responses from PUFs.

Our approach to this problem involves duplicating another selector chain for a different reason than the 2-XOR Arbiter PUF, as shown in Figure 6. The duplicated selector chain is implemented in SLICEs that neighbor the original selector chain. Each signal through the same route in each selector chain competes with the other. The Double Arbiter PUF generates 2-bit responses *r*1 and *r*2, as shown in Figure 6. This duplication-based approach can escape the wiring problem, because the length of the duplicated wire is expected to be similar to that of the original wire, given the symmetric layout implemented on neighboring SLICEs.

The authors of [17] proposed a 2-1 Double Arbiter PUF, whose 1-bit response is generated by XORing 2-bit responses from a Double Arbiter PUF, as shown in Figure 7. The aim of the *N*-XOR Arbiter PUFs is to improve the unpredictability by XORing multiple responses. To render the response less predictable, we can increase the number of XORed responses from Double Arbiter PUFs. The authors of [17] proposed a 3-1 Double Arbiter PUF (the main purpose of [17] is to increase variety of responses among chips) that XORs six responses by implementing a third Arbiter PUF on the same chip, as shown in Figure 8. We discuss the unpredictability of its responses in Section 5, with evaluation results showing how different these responses are among Double Arbiter PUFs in Section 6.

## 4. Preliminaries of Our Experiments

### 4.1. Experimental Environment

In our experiment, 64-bit Arbiter PUFs (*i.e.*, where 64-bit challenges are available) were implemented on three Xilinx Virtex-5 FPGAs (XC5VLX30) [21]: FPGA A, FPGA B, and FPGA C. These FPGAs were set up on a side-channel attack standard evaluation board G-II (SASEBO G-II) [22], and we provided challenges and obtained responses through a RS-232C cable connected to the SASEBO G-II. Xilinx ISE 13.2 and Xilinx PlanAhead 13.2 were used for the logic synthesis and for the floorplanning, respectively. Part of floorplanning design for the 3-1 Double Arbiter PUF is illustrated in Figure 9. In addition, Table 1 details the placement of primitives on SLICEs for our experiments. The notations for the PUF components in the first column of Table 1 are defined in Figure 8.

### 4.2. Intrachip Variation

The main goal of this paper is to evaluate the efficiency of XORing responses from Arbiter PUFs on the same chip. If several pairs of XORed responses have the same value, most of XORed responses become 0s. Because it is easy to predict the XORed responses in this situation, the pairs of responses should be completely different. The intrachip variation metrics is calculated with the following procedure. First, we implement two Arbiter PUFs that generate two responses on the same chip. Second, we provide the PUFs with *N* randomly chosen challenges, and the pair of *N*-bit responses is generated. Third, we calculate the Hamming distance (HD) between the pair of responses. The intrachip variation is defined as the HD divided by the response bit length, *N*. Ideally, the intrachip variation is 50%. In our experiment, *N* = 5,000.

In order to confirm the potential of our duplication-based approach in terms of unpredictability, the intrachip variation for a Double Arbiter PUF was compared to that of a conventional Arbiter PUF. As the preliminary to this evaluation, we define *r*1 and *r*2 as two responses from two conventional Arbiter PUFs implemented on the same chip. As shown in the second column of Table 2, the intrachip variation of the conventional Arbiter PUF between *r*1 and *r*2 was approximately 5%, which is quite low. These results imply that two Arbiter PUFs on the same chip will generate the same responses with the probability of 95%. That is, 95% of the responses from 2-XOR Arbiter PUF will become 0s, because pairs with the same value are XORed. It is easy to predict such responses, even without machine learning. The intrachip variation of the Double Arbiter PUF was evaluated by calculating the HD between two responses *r*1 and *r*2 from a Double Arbiter PUF, as shown in Figure 6. Because the intrachip variation of the Double Arbiter PUF is much higher than that of the conventional Arbiter PUF, as shown in the third column of Table 2, we can see potential of 2-1 Double Arbiter PUF to enhance the unpredictability.

### 4.3. Machine-Learning Environment

The authors of [23] reported the results of a machine-learning attack based on a support vector machine (SVM). We used an implementation of SVM called SVM^light^ [24] as machine-learning software. Between 100 and 1,000 CRPs were obtained from the Arbiter PUFs on each FPGA, and they were used by the SVM as training samples. For test samples, 10,000 challenges were provided to the SVM, and its responses were evaluated according to the prediction rate. The training and test samples were chosen randomly. With each number of training samples, the prediction rate of the machine-learning attack was calculated as the average of five trials.

## 5. Evaluation of Tolerance to Machine-Learning Attacks

First, the machine-learning results from [18] are introduced in Table 3. Note that these values are the average of the results shown in Table 4. They evaluated conventional Arbiter PUFs, 2-1 Double Arbiter PUFs, and 3-1 Double Arbiter PUFs using 1,000 training samples and 10,000 test samples. As shown in Table 3, the prediction rate for the responses from the 3-1 Double Arbiter PUF was 57%, and this approximates a random guess (*i.e.*, 50%).

However, there are no results from *N*-XOR Arbiter PUFs designed as countermeasures to machine-learning attacks (the results from the *N*-XOR Arbiter PUFs are shown in Figures 11 and 12). In this section, we compare the 2-XOR Arbiter PUF with the 2-1 Double Arbiter PUF and the 3-XOR Arbiter PUF with the 3-1 Double Arbiter PUF. That is, each pair of PUFs has the same hardware cost. Further, because there are no results regarding a dependency on the number of training samples in [18], we evaluate the four PUFs, using between 100 and 1,000 training samples. According to the results from this evaluation and the intrachip variation (see Section 4.2), we can conclude that the Double Arbiter PUFs have more potential in terms of unpredictability. To confirm the effectiveness of XORing responses with the Double Arbiter PUFs, we developed and evaluated a 4-1 Double Arbiter PUF.

### 5.1. Challenge Model for Double Arbiter PUFs

This paper aims at increasing tolerance to machine-learning attacks with the general delay model described in [12] and introduced in Section 2.2. This section discusses the validity of such a model for Double Arbiter PUFs. To do so, we return to the delay model for conventional Arbiter PUFs outlined briefly in Section 2.  Figure 10 shows part of the Double Arbiter PUF, which has the same signal condition as Figure 3. Consider a pair of challenges, where one is randomly chosen and the other is 1-bit flipped. In the case of a Double Arbiter PUF, when a 1-bit flipped challenge is provided, it is exchanged through whichever signal is supplied to right or left SR-Latch, whether the dashed or solid line. Certainly, the influence of the 1-bit flipped challenge is not equivalent to that of a conventional Arbiter PUF. However, when the same pair is converted into model vectors, that is, an original vector and a 1-bit flipped vector, the pair of signals through the dashed or solid line with the original vector has a total delay time similar to that of the pair of signals with the 1-bit flipped vector. Therefore, we believe that this model is also valid for Double Arbiter PUFs. Further, our complementary experiments show that the prediction rate using this model is higher than the prediction rate from using unconverted challenges.

It seems that the model for a Double Arbiter PUF requires twice as many parameters as there are additional selector chains. There is, however, no reason to introduce new delay parameters additionally to the conventional model since it is natural to assume that the delay parameters for two duplicated selector chains have identical properties.

### 5.2. 2-XOR Arbiter PUF versus 2-1 Double Arbiter PUF

The results from the machine-learning attack are shown in Figure 11. Only 100 training samples were needed to predict 10,000 responses from the 2-XOR Arbiter PUFs on all FPGAs, with approximately 95% probability. This is because 95% of the responses were 0s, as explained in Section 4.2 and Table 2.

Although the prediction rate for the 2-1 Double Arbiter PUF with few training samples appears to be low, 80% of the responses from the 2-1 Double Arbiter PUF on FPGA A with 1,000 training samples could be predicted, as shown in Figure 11(a). We cannot exclude the possibility that an attacker might predict the responses with even higher probability. According to the intrachip variation of the Double Arbiter PUF on FPGA B shown in the third column of Table 2, approximately 70% of the responses were 0s. Thus, approximately 70% of these responses could be predicted on FPGA B, regardless of the number of training samples, as seen in Figure 11(b). As implied by these results, the general delay model proposed in [12] can predict most of the responses from Double Arbiter PUFs. However, we can see the potential of the 2-1 Double Arbiter PUF in terms of unpredictability, because the prediction rate on FPGA C with 1,000 training data was approximately 57%, as shown in Figure 11(c), and because the tbl2-chip variation with the Double Arbiter PUF was high, as described in Section 4.2 with Table 2.

### 5.3. 3-XOR Arbiter PUF versus 3-1 Double Arbiter PUF

In order to enhance the effectiveness of XORing responses with our duplication-based approach, we can increase the number of XORed responses. The machine-learning attack results from the 3-XOR Arbiter PUF and the 3-1 Double Arbiter PUF are shown in Figure 12. The prediction rate of responses from the 3-XOR Arbiter PUF on all FPGAs increased with more training samples. Approximately 85% of the responses could still be predicted on all FPGAs. By contrast, even if an attacker obtained 1,000 training samples, it would be difficult to predict the responses from the 3-1 Double Arbiter PUF, because its prediction rate comes close to 50% (*i.e.*, random guess). The unpredictability of the 3-1 Double Arbiter PUF improved drastically, when compared to the 2-1 Double Arbiter PUF. It is true that the large number of PUF instances is preferable for determining the general properties of PUFs. However, considering the purpose of this paper, which is to enhance unpredictability, could be confirmed to some extent even with three FPGAs since the machine-learning attack for measuring the unpredictability is performed on each FPGA in our experiments.

### 5.4. 4-1 Double Arbiter PUF

In order to judge the effect of increasing the number of XORed responses, we developed a 4-1 Double Arbiter PUF with a fourth selector chain, as shown in Figure 13. Figure 12 includes the machine-learning attack results for this 4-1 Double Arbiter PUF. As shown in Figure 12, the tolerance of the 4-1 Double Arbiter PUF did not increase, and its results were comparable to the 3-1 Double Arbiter PUF. In Section 6, we compare the 3-1 Double Arbiter PUF with the 4-1 Double Arbiter PUF, using other metrics (as discussed in Section 5.1, it is easy to predict that most of the responses from the 4-XOR Arbiter PUF will be 0, because the number of XORed responses is an even number).

## 6. Overall Evaluation of the Conventional *N*-XOR Arbiter PUF and the *N*-1 Double Arbiter PUF

Previous work reported in [25, 26] suggests that the conventional Arbiter PUF on a Xilinx Virtex-5/Kintex-7/Artix-7 FPGA generates responses that are not particularly unique. The *N*-XOR Arbiter PUF [19] was designed not only to improve the unpredictability, but also to increase this uniqueness. Further, the Double Arbiter PUFs introduced in Section 3 were originally proposed as a technique for improving the uniqueness [16]. This section provides an overall evaluation of these PUFs that includes an evaluation of the uniqueness [17]. That is, our evaluation establishes which PUF performs best in terms of device authentication. The same FPGAs mentioned in Section 4.1 were used for this experiment:* namely*, FPGA A, FPGA B, and FPGA C. First, we provide a summary of the machine-learning attack results, using 1,000 training samples and 10,000 test samples (see Table 4). The additional metrics are defined in the following section.

### 6.1. Other Metrics for the Overall Evaluation

#### 6.1.1. Uniqueness

When the same challenge is given to the PUFs on different chips, their responses should be completely different. We evaluated this requirement by using the metric of uniqueness, which is calculated as follows. When we provide *N* randomly chosen challenges to PUFs on two chips, the pair of *N*-bit responses is generated, and we calculate the HD between the pairs of responses. The uniqueness is defined as the HD divided by the response bit length, *N*. Ideally, the uniqueness is 50%. In our experiment, *N* = 5,000.

#### 6.1.2. Randomness

One metric to measure the randomness of the responses is to analyze the proportion of 1s to 0s in the responses from a PUF, which should almost be the same when randomly chosen challenges are provided. In our experiment, we counted the number of 1s in the responses that were generated from a PUF when 2^16^ randomly chosen challenges were provided. The randomness is defined as this number divided by the response bit length, 2^16^. Again, the ideal randomness is 50% (the authors of [25] refer to this metric as* uniformity*).

#### 6.1.3. Steadiness

When the same challenges are provided to the same PUF on the same chip, the responses should have the same value. We evaluated this requirement by using a metric for steadiness, calculated as follows. The same *N* challenges are repeatedly given to the same PUF *M* times, and the average HD between two arbitrary *N*-bit responses out of *M* *N*-bit responses is calculated. The steadiness is defined as this average divided by response bit length, *N*. Ideally, the steadiness is 0%. In our experiment, *N* = 128 and *M* = 128 (the authors of [25] refer to this metric as* reliability*).

#### 6.1.4. Cost

It is also important to evaluate the hardware cost of the PUFs. We evaluated the number of occupied SLICEs during floorplanning. A lower cost is obviously better.

The uniqueness, randomness, and steadiness of the conventional Arbiter PUF, the 2-XOR Arbiter PUF, the 2-1 Double Arbiter PUF, the 3-XOR Arbiter PUF, and the 3-1 Double Arbiter PUF were introduced from [17] to the third, the fourth, and the fifth rows in Table 4, respectively. Note that the eighth column in Table 4 is newly introduced and provides the evaluation results for the 4-1 Double Arbiter PUF.

### 6.2. 2-XOR Arbiter PUF versus 2-1 Double Arbiter PUF

The uniqueness of the 2-XOR Arbiter PUF was slightly improved from that of the conventional Arbiter PUF, as shown in the third and fourth columns of Table 4. However, because the conventional Arbiter PUF has relatively low uniqueness, the 2-XOR Arbiter PUF whose 1-bit response is obtained by two XORing responses from two conventional Arbiter PUFs also generates responses with low uniqueness. By contrast, the uniqueness of the 2-1 Double Arbiter PUF was higher than that of the 2-XOR Arbiter PUF, as shown in the fourth and fifth columns of Table 4. It is clear that XORing responses from the Double Arbiter PUF are more effective than that from the conventional Arbiter PUF.

The randomness of the 2-XOR Arbiter PUF was considerably low, as shown in the fourth column of Table 4. This is because the intrachip variation was also low, since 1-bit responses generated by the two XORing responses become 0s, as discussed in Section 5.1. The randomness of the 2-1 Double Arbiter PUF was much higher than that of the 2-XOR Arbiter PUF, as shown in the fourth and fifth columns of Table 4.

The steadiness of the 2-XOR Arbiter PUF is approximately 1%, as shown in the fourth column of Table 4. We might say that the ideal steadiness is correlated with the low uniqueness of the 2-XOR Arbiter PUF that there is a trade-off between these two metrics. The steadiness of the 2-1 Double Arbiter PUF was around 10%, and this means that it is less stable than the 2-XOR Arbiter PUF, as shown in the fourth and fifth columns of Table 4. However, the steadiness of the 2-1 Double Arbiter PUF was comparable to that of the SRAM PUF and the Ring Oscillator PUF reported in [14].

### 6.3. 3-XOR Arbiter PUF versus 3-1 Double Arbiter PUF

The uniqueness of the 3-XOR Arbiter PUF was approximately 6%, as shown in the sixth column of Table 4, which means that the responses were almost as unique as those from the 2-XOR Arbiter PUF. By contrast, the uniqueness of the 3-1 Double Arbiter PUF was approximately 50%, as shown in the seventh column of Table 4, and this is an ideal result. We can conclude that the 3-1 Double Arbiter PUF utilizes XORing responses effectively.

The randomness of the 3-XOR Arbiter PUF was close to the ideal result, as shown in the sixth column of Table 4. This is because three responses (an odd number) were XORed with the conventional Arbiter PUF. The randomness of the 3-1 Double Arbiter PUF was almost ideal, as shown in the seventh column of Table 4, and this represented an improvement over the 2-1 Double Arbiter PUF.

The steadiness of the 3-XOR Arbiter PUF was approximately 1%, as shown in the sixth column of Table 4. This result is identical to that of the 2-XOR Arbiter PUF. The steadiness of the 3-1 Double Arbiter PUF was less than 15%, as shown in the seventh column of Table 4. The meaning of this result is discussed in next section.

### 6.4. 4-1 Double Arbiter PUF

We evaluated the 4-1 Double Arbiter PUF described in Section 5.3 using the above three metrics. The uniqueness and the randomness of the 4-1 Double Arbiter PUF were almost ideal, and these results were comparable to those of the 3-1 Double Arbiter PUF, as shown in the seventh and eighth columns of Table 4. However, the responses from the 4-1 Double Arbiter PUF were less stable than those from the 3-1 Double Arbiter PUF. The authors of [27] demonstrated that when the bit-error probability (*i.e.*, the steadiness) of a response is less than 15%, the response can be corrected using error-correcting code with a high level of probability. Because the steadiness of the 3-1 Double Arbiter PUF was less than 15%, we conclude that the 3-1 Double Arbiter PUF outperformed all other PUF-based authentication.

## 7. Conclusion

This paper introduced a new Arbiter PUF, called the Double Arbiter PUF, for enhancing the unpredictability of its responses. First, we evaluated the tolerance of the Double Arbiter PUFs to machine-learning attacks and compared it with the *N*-XOR Arbiter PUF, a well-known countermeasure against such machine-learning attacks. Our results showed that 85% of the responses from the conventional 3-XOR Arbiter PUF could be predicted with machine learning. By contrast, a 3-1 Double Arbiter PUF resulted in a prediction rate of 57%, which is close to 50% (a random guess). Second, we provided an overall evaluation of *N*-XOR Arbiter PUFs and *N*-1 Double Arbiter PUFs. We evaluated these approaches using metrics for the uniqueness, randomness, and steadiness, and we provided a comprehensive discussion of the results. The uniqueness of the 3-1 Double Arbiter PUF was almost ideal (50%), whereas that of the conventional 3-XOR Arbiter PUFs was approximately 6%. Further, we designed a 4-1 Double Arbiter PUF and evaluated it using the same metrics. Although its tolerance and uniqueness were almost the same as the 3-1 Double Arbiter PUF, the 4-1 Double Arbiter PUF was less stable than the 3-1 Double Arbiter PUF. Consequently, the 3-1 Double Arbiter PUF archived the best performance overall. However, the best parameter *N* for the *N*-1 Double Arbiter PUF might depend on the implementation platform or the PUF method. The PUF designer must carefully select optimal parameters in order to ensure the best performance.

## Figures and Tables

**Figure 1:** Structure of the Arbiter PUF.

**Figure 2:** Machine-learning attack against an Arbiter PUF.

**Figure 3:** Relationship between the challenge and model.

**Figure 4:** Structure of the 2-XOR Arbiter PUF.

**Figure 5:** Structure of the 3-XOR Arbiter PUF.

**Figure 6:** Structure of the Double Arbiter PUF.

**Figure 7:** Structure of the 2-1 Double Arbiter PUF.

**Figure 8:** Structure of the 3-1 Double Arbiter PUF.

**Figure 9:** Design of the 3-1 Double Arbiter PUF on Xilinx Virtex-5 FPGA. SR-Latches as Arbiters are fabricated by pairing the NAND with LookUp Table (LUT).

**Figure 10:** The challenge model for the Double Arbiter PUF.

**Figure 11:** Prediction rates of 2-XOR Arbiter PUF and 2-1 Double Arbiter PUF.

**Figure 12:** Prediction rates of 3-XOR Arbiter PUF and 3-1 and 4-1 Double Arbiter PUF.

**Figure 13:** Structure of the 4-1 Double Arbiter PUF.

**Table 1:** Placement of primitives on SLICEs for 3-1 Double Arbiter PUF. The value for the variable *j* can range from 0 to 63.

Descriptions		Primitives	SLICEs
(MUX_1L_(*j*), MUX_1R_(*j*))		F7BMUX	(SLICE_X14Y(76−*j*), SLICE_X15Y(76−*j*))
(MUX_2L_(*j*), MUX_2R_(*j*))			(SLICE_X16Y(76−*j*), SLICE_X17Y(76−*j*))
(MUX_3L_(*j*), MUX_3R_(*j*))			(SLICE_X18Y(76−*j*), SLICE_X19Y(76−*j*))
(MUX_4L_(*j*), MUX_4R_(*j*))			(SLICE_X20Y(76−*j*), SLICE_X21Y(76−*j*))

Pair of NAND in	SR-Latch_1	C6LUT	(SLICE_X14Y12, SLICE_X16Y12)
	SR-Latch_2		(SLICE_X16Y11, SLICE_X18Y11)
	SR-Latch_3		(SLICE_X18Y10, SLICE_X14Y10)
	SR-Latch_4		(SLICE_X15Y12, SLICE_X17Y12)
	SR-Latch_5		(SLICE_X17Y11, SLICE_X19Y11)
	SR-Latch_6		(SLICE_X19Y10, SLICE_X15Y10)

**Table 2:** Intrachip variation [%] of Arbiter PUF and Double Arbiter PUF.

FPGA	Arbiter PUF	Double Arbiter PUF
A	5.34	55.62
B	4.82	32.66
C	4.92	50.60

**Table 3:** Evaluation results of Arbiter PUF, 2-1 Double Arbiter PUF, and 3-1 Double Arbiter PUF.

Indicators	Arbiter PUF	2-1 Double Arbiter PUF	3-1 Double Arbiter PUF	Ideal
Pred. rate [%]	86.3^†^	69.0^†^	57.0^†^	50
Cost (ratio)	1	2	3	—

^†^These values are introduced from [18].

**Table 4:** Results of the overall evaluation.

Metrics	FPGA	Conventional Arbiter PUF	2-XOR Arbiter PUF	2-1 Double Arbiter PUF	3-XOR Arbiter PUF	3-1 Double Arbiter PUF	4-1 Double Arbiter PUF	Ideal
Prediction rate [%] (with 1000 training data)	A	86.32^^†^^	93.50	80.72^†^	85.82	56.47^†^	56.11	50
	B	86.36^†^	95.28	69.52^†^	85.95	57.45^†^	55.60	
	C	86.30^†^	95.41	56.64^†^	85.25	56.75^†^	54.73	

Uniqueness [%]	A with B	4.72^‡^	4.96^‡^	41.36^‡^	5.96^‡^	50.60^‡^	50.46	50
	B with C	4.96^^‡^^	5.62^‡^	49.70^‡^	6.76^‡^	51.34^‡^	49.86	
	C with A	4.44^‡^	5.58^‡^	48.06^‡^	6.32^‡^	48.78^‡^	49.76	

Randomness [%]	A	53.81^‡^	6.32^‡^	55.19^‡^	54.88^‡^	55.68^‡^	55.67	50
	B	56.53^‡^	4.72^‡^	31.40^‡^	55.05^‡^	52.54^‡^	54.76	
	C	54.00^‡^	4.93^‡^	50.63^‡^	54.96^‡^	53.59^‡^	54.59	

Steadiness [%]	A	0.76^‡^	1.43^‡^	7.79^‡^	1.43^‡^	14.11^‡^	34.96	0
	B	0.83^‡^	1.36^‡^	11.22^‡^	1.36^‡^	10.93^‡^	18.99	
	C	0.45^‡^	0.52^‡^	10.05^‡^	0.74^‡^	10.35^‡^	25.85	

Cost (# of SLICEs)	—	177^*∗*^	299	303^*∗*^	426	436^*∗*^	577	—

^†^These values are introduced from [17].

^‡^The results of [18] shown in Table 3 are the averages of these values.

^*∗*^These values are introduced from [18].
